# A Cautionary Tale of a Complex Peri-Trochanteric Fracture in a Very Important Person (VIP) Patient at a Community-Based Hospital: A Case Report

This article has been retracted.

**DOI:** 10.7759/cureus.33150

**Published:** 2022-12-30

**Authors:** Jason P Den Haese, Blake E Delgadillo, Bryan G Anderson, Shawn W Storm

**Affiliations:** 1 Department of Orthopedic Surgery, Lake Erie College of Osteopathic Medicine (LECOM) Health, Millcreek Community Hospital, Erie, USA; 2 Department of Orthopedic Surgery, Lake Erie College of Osteopathic Medicine (LECOM), Bradenton, USA; 3 Department of Spine Surgery, Swedish Neuroscience Institute, Seattle, USA

**Keywords:** hip arthroplasty, cephalomedullary nail, hip fracture, peritrochanteric fracture, intertrochanteric fracture

## Abstract

Peri-trochanteric fractures with an extension into the femoral neck are relatively rare. Due to the lack of a defined treatment in the literature, these fractures pose a challenge to orthopedic surgeons. This case report highlights the value of timing to surgical intervention, choosing the appropriate operative course, not treating very important person (VIP) patients differently than standard patients, and decreasing unnecessary costs for the patient and the US healthcare system.

An 85-year-old male VIP patient presented to the emergency department (ED) with a left peri-trochanteric fracture with an extension into the ipsilateral femoral neck. The initial plan was to perform arthroplasty with diaphyseal fixation. However, the community-based hospital would have to wait two to three days for the proper implants, and the patient insisted on being treated at this hospital. Due to concerns about increased mortality with delayed treatment, the patient underwent short cephalomedullary nail (CMN) fixation the next day. On postoperative day (POD) 49, a *pop* was heard and felt while ambulating, and radiographs revealed substantial lateral cutout of the CMN and subsidence of the femoral head. On POD 54, the patient underwent a successful left total hip arthroplasty using a modular diaphyseal press-fit femoral component, which resulted in an uneventful recovery.

This case illustrates a cautionary tale in choosing the appropriate operative course for a VIP patient with a peri-trochanteric fracture extending into the femoral neck (a relatively rare fracture type that has no clearly defined treatment option). This is imperative to reduce pain and length of stay for the patient, postoperative complications, and cost. Based on the results from the second procedure and weighing the risk of prolonged treatment, the authors believe that this patient would likely have benefited from a primary arthroplasty procedure given his body habitus and complex fracture pattern.

## Introduction

The region between the greater and lesser trochanter composed of dense trabecular bone is known as the intertrochanteric (IT) region of the femur [1]. IT fractures, defined as fractures that involve the proximal portion of the femur in the IT region, rank as the most prevalent type of extracapsular fracture of the proximal femur [2,3]. Among this common fracture type, it should be noted that a peri-trochanteric fracture with an extension into the ipsilateral femoral neck is relatively rare, with considerably few cases reported since 1989 [4-6]. A chronic disease that involves bone loss, such as diabetes mellitus, Cushing’s syndrome, hyperthyroidism, and hyperparathyroidism, is associated with a two- to sevenfold increase in hip fracture risk [2]. In the geriatric population, unstable IT fractures are common [7].

The treatment of IT fractures has become an issue of health resources; of all surgically treated fractures, IT fractures show the highest postoperative fatality rate [2]. Accounting for 44% of all hip fracture costs, IT fractures typically cost US$52,512 per patient, which coincides with a US$2.63 billion economic burden on the U.S. healthcare system [8]. Although the current standard of care for fixation or arthroplasty of hip fractures is 24 to 48 hours after injury, operative courses can be delayed for a variety of reasons [9]. Conservative surgical intervention should be avoided [10]. Early surgical intervention and choosing the appropriate operative course can result in decreased pain, shortened length of stay, and fewer complications [9]. Treatment of IT fractures can be further complicated in a very important person (VIP) patient. This can be defined as those who hold celebrity status, power, or perceived connections [11]. *VIP syndrome* results in a vicious cycle of less-than-ideal clinical judgment, with attempts to meet unrealistic patient demands, which results in suboptimal outcomes. VIP patients often have demands that can cause medical providers to steer away from the standard of care [11].

The purpose of this case study is to evaluate the timing of surgical intervention, choice of surgical treatment, and complications associated with surgical treatment in a VIP patient with a comminuted peri-trochanteric fracture extending into the femoral neck.

## Case presentation

An 85-year-old male, who was considered to be a VIP patient by the hospital staff, presented to the emergency department (ED) after sustaining a mechanical fall while ambulating in his home. The patient landed on his left hip, and he was unable to rise from the floor using his strength due to left hip pain. An ED physician evaluated him and identified a left hip fracture via physical exam and appropriate imaging (Figures 1-4). No other injuries were identified at that time. The patient was admitted, and the orthopedic team was consulted to manage the hip fracture.

**Figure 1:** (A) An anteroposterior pelvis radiograph demonstrating a comminuted left peri-trochanteric femur fracture extending into the femoral neck. Previous right total hip arthroplasty and a penile implant can also be visualized. (B) A left hip anteroposterior radiograph with traction to better appreciate the fracture line. (C) A magnified view of the left hip anteroposterior hip radiograph with traction demonstrating the same fracture pattern stated previously.

**Figure 2:** (A) An anteroposterior radiograph of the left femur revealing no subtrochanteric extension of the peri-trochanteric femur fracture or previous orthopedic hardware present. (B) An anteroposterior radiograph of the left knee and (C) a lateral radiograph of left knee revealing severe left knee osteoarthritis without previous orthopedic hardware present.

**Figure 3:** (A) and (B) Two different slices of an axial view CT of the left hip and (C) a coronal view CT of the left hip revealing a comminuted left peri-trochanteric femur fracture extending into the femoral neck. CT, computed tomography

**Figure 4:** (A) and (B) Two 3D-reconstructed CT views of the left hip revealing a comminuted left peri-trochanteric femur fracture extending into the femoral neck. CT, computed tomographic

The patient’s past medical history revealed hypertension, gastroesophageal reflux, morbid obesity, and left knee osteoarthritis. The patient used a cane to ambulate at baseline due to chronic left knee pain. Upon reviewing all systems, the only complaint expressed was the patient’s left hip pain. Past surgical history included right total hip arthroplasty (THA), right hemicolectomy, bilateral inguinal herniorrhaphy, laparoscopic lysis of adhesions due to small bowel obstruction, and a penile implant.

The patient’s vital signs were stable, and he was afebrile. The patient had a body mass index (BMI) of 40.1. On examination, the left lower extremity was shortened and externally rotated with pink skin and no lesions. All compartments were soft and compressible. The patient had pain over his greater trochanter with palpation, pain that radiated to the left groin with log roll, and severe pain with any range of motion. The patient was distally neurovascularly intact. No injury or deformity was identified for the right lower extremity and bilateral upper extremities.

The orthopedic attending on call decided to proceed with closed versus open reduction and internal fixation of the fracture with a short cephalomedullary nail (CMN) the next day.

At the time of surgery, the patient was prepped and draped in a normal fashion. The patient was placed in supine positioning without abduction of the torso, and anatomic closed reduction was obtained with traction, internal rotation, and adduction of the left hip. A longitudinal lateral incision proximal to the greater trochanter and in line with the femur was made. The guidewire was passed [12]. However, given the large body habitus of the patient, the opening reamer was not able to be passed over the guidewire due to the abdominal/flank pannus. After much difficulty and time trying to get the opening reamer introduced to the wound, intraoperative repositioning of the lower left extremity with hip adduction was made to improve further instrument access to the proximal femur [12]. This change in hip positioning resulted in the loss of anatomic reduction of the fracture and resultant varus positioning at the fracture site. The instrumentation was placed uneventfully, albeit not in an ideal position, given the varus position of the fracture site, and the case concluded uneventfully. Plain radiographs were obtained on postoperative days (PODs) 0, 14, and 30 (Figure 5).

**Figure 5:** (A) An anteroposterior radiograph of the left hip and an oblique radiograph of the left hip on postoperative day 0. (B) An anteroposterior radiograph of the left hip and an oblique radiograph view of the left hip on postoperative day 14 revealing a controlled collapse of the femoral head and neck along the cephalomedullary nail without evidence of implant failure or cutout. (C) An anteroposterior radiograph of the left hip and an oblique radiograph of the left hip on postoperative day 30 revealing a further controlled collapse of the femoral head and neck along the cephalomedullary nail without evidence of implant failure or cutout.

At the time of this index surgery, the following items were used: TFN-ADVANCED^TM^ Proximal Femoral Nailing Advanced System (TFNA, DePuy-Synthes, Raynham, MA, USA); 130°, 10 mm × 170 mm nail; 110 mm helical blades; and 40 mm distal locking screws. The total operating room (OR) time was 2.5 hours. The estimated blood loss was 400 cc.

Given the malpositioning of the fracture site and suboptimal placement of the hardware, the patient was limited to toe-touch weight bearing of the left lower extremity with the assistance of a rolling walker for seven weeks due to concern about implant cutout. The patient was discharged to an inpatient rehabilitation center on POD 2. On POD 47, radiographs were obtained demonstrating the healing of the fracture. Thus, the patient was made weight-bearing as tolerated and subsequently discharged home from inpatient rehabilitation.

On POD 49, the patient re-presented to the ED after he felt and heard a loud *pop* in his left hip while ambulating in his home. Imaging was obtained (Figure 6), and the orthopedic index surgeon was consulted. Due to the complex nature of the possible revision surgery needed, the decision was made to transfer the patient to a tertiary center where an orthopedic trauma and reconstruction fellowship-trained surgeon could undertake revision surgery. The transfer was made on POD 52. The patient underwent a successful left THA on POD 54 using a modular diaphyseal press-fit femoral component. The patient was made weight-bearing as tolerated immediately after his revision surgery. On POD 56 or POD 2, the patient was transferred back to his previous inpatient rehabilitation facility. Plain radiographs were obtained on POD 71 from primary surgery or POD 14 from revision surgery (Figure 7), demonstrating uncomplicated THA without evidence of fracture or loosening. Now, three years later, the patient’s postoperative course has continued to progress without any complications or complaints of pain or limited mobility.

**Figure 6:** (A) An anteroposterior radiograph of the pelvis, (B) an anteroposterior radiograph of the left hip, and (C) a cross-table lateral radiograph of the left hip on postoperative day 49 revealing substantial lateral cutout of cephalomedullary nail and subsidence of the femoral head.

**Figure 7:** (A) An anteroposterior radiograph of the pelvis, (B) an anteroposterior radiograph of the left hip, and (C) a cross-table lateral radiograph of the left hip on POD 71 (from the primary procedure) or POD 14 (from revision procedure) revealing a left total hip arthroplasty using a calcar replacing the modular femoral component with a diaphyseal press-fit stem. POD, postoperative day

## Discussion

Hip fractures are fairly common among the elderly population, and the injuries carry a mortality rate of 5% to 10% at one month and 12% to 27% at one year from surgery. The literature supports that patients who undergo early surgical intervention have a significantly lower risk of death [10]. IT fractures require prompt surgical intervention; the current standard of care for fixation or arthroplasty of hip fractures is within 24 to 48 hours of hospitalization [9]. Furthermore, Maheshwari et al. found that every 10-hour delay from hospital admission to surgery demonstrates a 5% increase in the odds of one-year mortality [13].

In this case, the patient was diagnosed with a comminuted peri-trochanteric femur fracture extending into the femoral neck (Figures 1-4). Multiple discussions were held among the orthopedic team members, which included an intern resident, a chief resident, and a fellowship-trained orthopedic surgeon. In these conversations, consideration was given to operative fixation versus arthroplasty using a short CMN, long CMN, hemiarthroplasty using a diaphyseal fixation prosthesis, or a THA using a diaphyseal fixation prosthesis. Unfortunately, this fracture occurred on the weekend, and due to this community-based hospital’s limited supply, it would have taken approximately 48 to 72 hours for the hospital to receive the proper arthroplasty implants. Although the orthopedic team’s first choice was a diaphyseal press-fit hemiarthroplasty, they ultimately chose to proceed with a short CMN within 24 hours of injury due to concerns for increased risk of complications and mortality with significantly delayed treatment [9,10,13]. Additionally, the VIP patient insisted on being treated at this hospital as soon as possible, and he likely would not have held the same status at another hospital, which could have led to further delayed transfer time. This patient’s combined comminuted peri-trochanteric femur fracture with femoral neck fracture extension pattern is a relatively rare type that has no clearly defined treatment option [3,14]. There is evidence that treatment with a CMN can be effective in these fracture types. Yoo et al. attempted to classify this fracture and showed that 33 patients of a similar age and fracture type had an 85% bone union rate with a CMN (noting that every failed union correlated with an unsatisfactory reduction on the postoperative lateral plain film views) [3]. In addition to this case, there is evidence in the literature of successful treatment with arthroplasty [15].

VIP patients are defined as those who possess large amounts of wealth or prestige. VIP patients, like in this case, can instill fear and nervousness in medical providers, which can lead to suboptimal treatment and even worse medical outcomes [16]. Medical professionals must do their best to adhere to the standard of care for the treatment of VIP patients, even if it means not perfectly adhering to their wishes. When dealing with any patient, it is often difficult to choose the best operative course if no treatment method is noted in the current literature. This added to the difficult decision-making in this case, beyond the sheer timing outlined previously.

One of the main complications of CMN fixation is cutout, which is defined as the femoral head and neck intramedullary implant perforating through the superior posterolateral cortex of the femoral neck/head followed by rotation and varus collapse of the head-neck fragment [17]. This patient experienced a significant cutout of the nail, which resulted in a revision to a THA with a modular diaphyseal press-fit component (Figures 5-7). This may have resulted from insufficient presurgical torso abduction positioning of this morbidly obese patient on the fracture table, leading to an inability to gain optimal access to the proximal femur starting point, which required intraoperative manipulation of the operative extremity and loss of fracture reduction. Subsequent fracture fixation at the time of the index surgery was completed in a varus position, ultimately leading to fixation failure on POD 47.

As noted previously, IT fractures account for 44% of all hip fracture costs; the average cost is US$52,512 per patient and an astonishing US$2.63 billion economic burden on the U.S. healthcare system [8]. In this patient’s case, the cost was even higher due to the requirement of multiple procedures in a relatively short period.

The orthopedic team choosing an operative course with CMN fixation led the patient to endure two months of physical therapy (PT) just to be followed up by another operation, which was again followed by more PT. As a major learning point, the authors understand the morbidity and mortality of waiting more than 48 hours to operate on the proximal femur [9,10,13]; however, in retrospect, they believe that waiting to use the arthroplasty implants at the time of the index procedure would have prevented unnecessary rehabilitation and second surgery. Another option would have been to refer the patient to a hospital that was able to perform arthroplasty within the appropriate time frame. However, the authors acknowledge the additional delayed surgical time that the patient would have accrued with a transfer to another facility. Furthermore, given the patient’s VIP status, the patient and his family wanted the earliest possible surgery to be performed at the institution he was accustomed to. It is also noteworthy that the patient had a list of problems with the short CMN fixation, including lateral cutout, subsiding of the femoral head, and increasing tip-to-apex distance (Figures 5-6). After undergoing a left THA using a calcar replacing the modular femoral component with a diaphyseal press-fit stem on POD 54 (from the first procedure), the patient was able to bear weight as tolerated immediately after surgery. From this point on, the patient’s recovery was uncomplicated, which we project would have been the case if the arthroplasty was performed upon admission to the hospital in this patient with a large body habitus and complex peri-trochanteric fracture pattern.

Early surgical intervention and choosing the appropriate operative course can result in decreased pain, shortened length of stay, and fewer complications [9]. Patients, whether they are VIPs or not, deserve to be treated with the best care possible. The purpose of this case study was to highlight the learning points that future orthopedic teams can use to prevent similar cases from happening. Although the treatment of choice is debated in the literature [3,14], we believe that the correct primary procedure for this patient would have been arthroplasty. This choice is based on the high likelihood of CMN failure with the difficult patient positioning and complex fracture pattern. These learning points, as described previously, include the timing of surgical intervention, choosing the appropriate operative course, not treating VIP patients any differently than standard patients, and decreasing unnecessary costs for the patient and the U.S. healthcare system. 

## Conclusions

This case illustrates a cautionary tale in choosing the appropriate operative course for a VIP patient with a peri-trochanteric fracture extending into the femoral neck (a relatively rare fracture type that has no clearly defined treatment option). This is imperative to reduce patient pain and length of stay, postoperative complications, and cost. Based on the results from the second procedure and weighing the risk of prolonged treatment, the authors believe that this patient would likely have benefited from a primary arthroplasty procedure given his large body habitus and complex fracture pattern. 
